# Celiac disease in pediatric patients according to HLA genetic risk classes: a retrospective observational study

**DOI:** 10.1186/s13052-021-01052-1

**Published:** 2021-05-05

**Authors:** Carlo Tolone, Marisa Piccirillo, Pasquale Dolce, Salvatore Alfiero, Mattia Arenella, Marina Sarnataro, Patrizia Iardino, Alessia Pucciarelli, Caterina Strisciuglio

**Affiliations:** 1 Department of Pediatrics, University of Campania Luigi Vanvitelli, Naples, Italy; 2 Department of Public Health, University of Naples Federico II, Naples, Italy; 3 UOC Clinic and Molecular Pathology, University of Campania Luigi Vanvitelli, Naples, Italy; 4 Department of Precision Medicine, University of Campania Luigi Vanvitelli, Naples, Italy

**Keywords:** Celiac disease, HLA-DQ_2/_ DQ_8_, Clinical and serological manifestation

## Abstract

**Background:**

Celiac disease (CD) is an autoimmune enteropathy in which HLA-DQ haplotypes define susceptibility. Our aim was to evaluate if belonging to a certain HLA-DQ class risk could be associated to the clinical, serological and histological presentation of CD.

**Methods:**

We performed a retrospective observational monocentric study including all 300 patients diagnosed with CD, who underwent HLA typing. Clinical, serological and histological data was collected from clinical records and their association with HLA-DQ class risk was verified through statistical tests.

**Results:**

In our sample mean age at onset was 6.7 ± 4.2 years, with a prevalence of females (*n* = 183; 61%), typical symptoms (*n* = 242; 80.6%) and anti-tTG IgA ≥ 100 U/mL (*n* = 194; 64.7%). Family history was present only in 19% (*n* = 57) of patients, and it was not significantly associated with any of the clinical and demographical data analyzed or the belonging to a certain HLA-DQ class risk. We found in the male population more frequently a coexistence of CD and atopic syndrome (males: *n* = 47; 40.2%; females: *n* = 50; 27.3%; *p* = 0.020).

Early age of onset, instead, was associated with typical symptoms (*m* = 6.4 ± 4; *p* = 0.045) and elevated liver enzymes (*m* = 5 ± 3.8; *p* < 0.001), while later age of onset was associated with presence of other autoimmune diseases (*m* = 8.2 ± 4; *p* = 0.01).

We observed statistically significant influences of HLA class risk on antibodies and liver enzymes levels: G1, G4 and G2 classes showed more frequently anti-tTG IgA ≥ 100 U/mL (*n* = 44; 80%, *n* = 16; 69.6%, *n* = 48; 67.6% respectively; *p*-value = 0.037), and in patients from G2 class we found enhanced liver enzymes (*n* = 28; 39.4%; p-value = 0.005). HLA class risk was still significantly associated with anti-tTG ≥ 100 (*p* = 0.044) and with hypertransaminasemia (*p* = 0.010) after a multiple logistic regression adjusted for the effect of gender, age at onset and family history.

**Conclusions:**

We failed to prove an association between HLA-DQ genotypes and the clinical features in our CD pediatric patients. Although, our results suggest an effect of the DQB1–02 allele not only on the level of antibodies to tTG, but possibly also on liver involvement.

## Background

Coeliac disease is an immune-mediated systemic disorder triggered by the consumption of gluten, a storage protein complex contained in some cereals (e.g. wheat, barley, rye) [1]. The ingestion of gluten, in genetically susceptible individuals, causes a chronic inflammatory process in the small intestine resulting in malabsorption.

According to recent epidemiological studies, the prevalence in the Western countries has been estimated to be around 1%. More than 600.000 celiac patients live in Italy and around 500 new diagnoses are made every year, although it seems that for every diagnosed celiac patient another 5 patients are undiagnosed.

Nowadays, CD is more common between the ages of 19 and 40, with a male-female ratio of 1:2 [2].

A fundamental role in the pathogenic pathway is played by genetic susceptibility, determined by major histocompatibility complex class II molecules, especially HLA-DQ2 and HLA-DQ8 antigens. Approximately, 85% of celiac patients possesses at least one copy of HLA-DQ2, 5–10% one copy of HLA-DQ8 and less than 5% just a half of the heterodimer DQ2, more often DQB1*02 [3, 4].

An important dose effect has been recognized for the glycoprotein DQ2 that, when possessed in double dose, enhances the chances of developing CD, because HLA’s ability of interact with gliadin specific peptides and stimulate lymphocytes is doubled [5].

The α and β chains of DQ2 molecules are encoded by the HLA-DQA1*0501-DQB1*0201 and the DQA1*0301-DQB1*0302 alleles, that confer the essential genetic susceptibility to develop the disease. DQ2 and DQ8 heterodimers are able to bind gliadin peptides, creating an HLA-antigen complex that can be recognized by CD4+ T lymphocytes in the intestinal mucosa, with the release of pro-inflammatory cytokines responsible for the chronic inflammation and histological damage [6].

Celiac disease is characterized by extremely heterogeneous symptoms, e.g. it can appear in a typical presentation with gastrointestinal complaints or in a non-classical form with iron deficiency anemia, hypertransaminasemia, short stature, asthenia. Frequently, CD can be associated with other autoimmune disease such as type I diabetes mellitus, autoimmune thyroid disease. or liver disease [7–10].

Diagnosis can be suspected when enhanced levels of disease-associated antibodies, including tissue transglutaminase antibodies (tTG), endomysium antibodies (EMA) and deamidated gliadin antibodies (DMG) are detected, but has to be confirmed through a duodenal biopsy showing lymphocyte invasion in the epithelium, hyperplasia of the crypts and various grades of villous atrophy. The severity of the histological lesions can categorize the intestinal damage in three stages, according to Marsh-Oberhuber classification [11].

These serological and histological manifestations have been used until recently to diagnose CD, however the 2012 European Society for Paediatric Gastroenterology Hepatology and Nutrition (ESPGHAN) guidelines indicated that a biopsy can be omitted in symptomatic children with: tTG IgA levels ≥100 U/mL (≥ 10 times the upper limit), positive EMA, and HLA risk haplotypes [12].

A stratification in five genetic risk classes (G1-G5), according to the presence of a particular HLA haplotype, has been suggested to value the real risk of developing CD among susceptible individuals [13].

It is unclear why patients show such a heterogeneity amount of signs and symptoms, and the aim of this observational retrospective study was to assess whether belonging to a specific genetic risk class may be associated with different clinical manifestations at the onset of CD.

## Materials and methods

### Study population

A total of 428 pediatric patients, aged less than 18 years, were diagnosed with CD according to the corresponding valid European Society for Paediatric Gastroenterology Hepatology and Nutrition (ESPGHAN) criteria [14] between 2010 and 2019 at the Pediatric Gastroenterology Department of University of Campania “Luigi Vanvitelli”. All 300 consecutive patients, who underwent HLA typing, were included in the study. All were children with Italian ancestry. Clinical data were obtained from medical files retrospectively by independent investigators, blinded to the HLA class risk of the patients. The study was reviewed and approved by the local medical ethics board (13,568/2020).

### Clinical characteristics

We considered the following variables: 1) sex; 2) age at onset, considering the time of first appearance of symptoms that could be explained by celiac disease; 3) family history of CD; 4) clinical presentation at diagnosis, classified as typical, meaning onset of gastrointestinal symptoms (chronic diarrhea, constipation, abdominal pain, lack of appetite, vomiting, abdominal distension associated with meteorism), weight loss or deficiency in weight gain, short stature or deficiency in height gain and non-typical, meaning iron deficiency anaemia, elevated liver enzymes (ALT > 36 mU/mL; AST > 29 mU/mL), headache, asthenia, joint pain and muscular pain, oral thrush, dermatitis herpetiformis or absence of symptoms; 4) serological results: IgA or IgG (in IgA deficient patients) anti-tTG and/or EMA, highlighting the study population with > 10 times the upper limit of normality in case of anti-tTG positivity; 5) histological lesions, according to the Marsh-Oberhuber classification [15]; 6) co-existence of autoimmune disease or atopic conditions.

### Genetics

Genotyping for celiac disease-associated HLA alleles was performed with the XeliGen XL (Eurospital SpA-Trieste) following the recommendations of the manufacturer [13, 16].

Haplotypes were categorized in five genetic risk classes: G1- (homozygous DR3-DQ2 genotype, with two copies of DQA1*05 and DQB1*02 genes; the heterozygous DR3/DR7 genotype, with one copy of DQA1*05 and two copies of DQB1*02); G2- (a single molecule of HLA-DQ2.2 and one copy of DQA1*05); G3- (the heterozygous DR3/DR5 genotype, characterized by two doses of DQA1*05 and one dose of DQB1*02); G4- (homozygous HLA-DQ8/DR4 or homozygous DQ2/DR7); G5 characterized by other molecules of HLA-DQ.

### Statistical analysis

Data were presented as frequency (percentage) for categorical variables and as mean ± standard deviation for quantitative variables.

The patients were divided in 5 groups according to the genetic risk classes. Subsequently, the differences among the 5 groups in terms of presence of diarrhea or constipation, absence of symptoms, anti-tTG IgA levels < or > 100 U/mL, elevated liver enzymes, co-existence of other auto-immune or atopic diseases were tested using the χ^2^ test or the Fisher’s exact test, as appropriate, for categorical variables and ANOVA or Kruskal Wallis Test, as appropriate, for quantitative variables.

Multiple logistic regressions were carried out to verify whether HLA class risk was significantly associated with the considered variables after adjusting for the effect of gender, Age at onset, and Family history.

All statistical analysis were performed also considering the sub-sample of 144 patients, who underwent duodenal biopsy.

Statistical analysis was performed using the R software for statistical computing. A *p*-value < 0.05 was considered as statistical significance.

## Results

Age at onset ranged from 7 months to 17 years in our 300 CD patients, with a mean of 6.7 ± 4.2 years. Of the total study population, 117 (39%) were males and 183 females (61%). All patients showed positive anti-tTG/EMA serology. Among the patients, the vast majority showed elevated anti-tTG IgA levels (64.7%) and symptoms (80.6%), therefore they were diagnosed according to the ESPGHAN 2012 criteria without biopsies. Only 144 patients underwent duodenal biopsy and severe villous lesion (Marsh 3b or 3c) was observed in 61.8% of the patients (Table 1). In this group we evaluated the association between HLA risk classes with family history, age at onset, presence of typical symptoms or absence of symptoms, autoimmune diseases, atopic syndrome, antibody and liver enzymes levels, but we did not find any statistically significant association. In this sample of 144 patients we also tested for any relation between sex, family history and age at onset with all the variables considered in the study, but we did not find any significant association.

**Table 1:** Clinical characteristics of enrolled patients

	Total *n* = 300
Male	117 (39%)
Age at onset	6.7 ± 4.2
Family history	57 (19%)
Lack of symptoms	38 (12.7%)
Typical GI symptoms^a^	242 (80.7%)
- Constipation	50 (16.7%)
- Diarrhea	111 (37%)
- Abdominal pain	71 (23.7%)
- Lack of appetite	72 (24%)
- Vomiting	44 (14.7%)
- Abdominal distension/meteorism	25 (8.3%)
- Weight loss	145 (48.3%)
- Short stature	62 (20.6%)
Non typical GI symptoms^a^	58 (19.3%)
- Iron deficiency anemia	138 (46%)
- Headache	15 (5%)
- Asthenia/joint or muscular pain	56 (18.7%)
- oral trush	28 (9.3%)
Anti-tTG ≥ 100	194 (64.7%)
AI disorders^b^	33 (11%)
Atopy	97 (32.3%)
Hypertransaminasemia	74 (24.7%)
Marsh 3b/3c^c^	89 (61.8%)

^a^*GI* Gastrointestinal

^b^*AI* Autoimmune

^c^Only 144 patients underwent duodenal biopsy

We explored the influence of sex and age on all the variables (Table 2). Although females outnumbered males, we didn’t find significant association with the variables explored. On the contrary we found in the male population more frequently a coexistence of CD and atopic syndrome (males: *n* = 47; 40.2%; females: *n* = 50; 27.3%), statistically significant (*p* = 0.020).

**Table 2:** Association between sex and clinical and serological variables

	Total n = 300	Male *n* = 117	Female *n* = 183	p-value
Family history	57 (19%)	22 (18.8%)	35 (19.1%)	0.899
Anti-tTG ≥ 100	194 (64.7%)	71 (60.7%)	123 (67.2%)	0.249
AI disorders^a^	33 (11%)	14 (12%)	24 (13.1%)	0.501
Atopy	97 (32.3%)	47 (40.2%)	50 (27.3%)	0.020
Hypertransaminasemia	74 (24.7%)	23 (19.7%)	51 (27.9%)	0.108
Marsh 3b/3c^b^	89 (61.8%)	34 (56.7%)	55 (65.5%)	0.283

^a^*AI* Autoimmune

^b^Only 144 patients underwent duodenal biopsy: 60 male and 84 female

Early age of onset, instead, was associated with typical symptoms (*m* = 6.4 ± 4 vs 7.6 ± 3.8; *p* = 0.045) and elevated liver enzymes (*m* = 5 ± 3.8 vs 7.1 ± 4.2; *p* < 0.001), while later age of onset was associated with the presence of other autoimmune diseases (*m* = 8.2 ± 4 vs 6.4 ± 4.1; *p* = 0.01) (Table 3).

**Table 3:** Association between age at onset and clinical and serological variables

	Presence	Absence	p-value
Lack of symptoms	7.5 ± 3.9	6.5 ± 4.2	0.162
Typical GI symptoms^a^	6.4 ± 4.2	7.6 ± 3.8	0.045
AI disorders^b^	8.2 ± 4.2	6.4 ± 4.1	0.010
Atopy	7.1 ± 4.3	6.4 ± 4.1	0.205
Hypertransaminasemia	5 ± 3.8	7.1 ± 4.1	0.000
Anti-tTG ≥ 100	6.7 ± 4.3	6.5 ± 4.0	0.756
Marsh 3b/3c^c^	6.6 ± 4.0	7 ± 4.1	0.751

(All the results in this table refer to mean age at onset±standard deviation)

^a^*GI* Gastrointestinal

^b^*AI* Autoimmune

^c^Only 144 patients underwent duodenal biopsy

Then we observed the influence of genotypes on the clinical and demographical variables of CD (Table 4). A family history of CD was observed in 57 patients (19%) and it was not significantly associated with any of the clinical and demographical data analyzed. Moreover, we didn’t find significant changes between family history across the risk classes (*p* = 0.265). Also, the association between sex and genotypes was not statistically significant (*p* = 0.366).

**Table 4:** Association between HLA class risk and clinical and serological variables (univariate analysis)

	Total n = 300	G1 *n* = 55	G2 *n* = 71	G3 *n* = 100	G4 *n* = 23	G5 *n* = 51	p-value
Male	117 (39%)	25 (45.5%)	21 (29.6%)	41 (41%)	8 (34.8%)	22 (43.1%)	0.364
Age at onset	6.7 ± 4.2	6.7 ± 4.5	6.2 ± 4.1	6.7 ± 4	8.5 ± 5.3	6.3 ± 3.8	0.235
Family history	57 (19%)	14 (25%)	12 (17%)	21 (21%)	1 (4.3%)	9 (18%)	0.265
Anti-tTG ≥ 100	194 (64.7%)	44 (80%)	48 (67.6%)	56 (56%)	16 (69.6%)	30 (58.8%)	0.037
AI disorders^a^	33 (11%)	6 (10.9%)	5 (7%)	12 (12%)	1 (4.3%)	9 (17.6%)	0.664
Atopy	97 (32.3%)	19 (34.5%)	19 (26.8%)	32 (32%)	8 (34.8%)	19 (37.3%)	0.779
Hypertransaminasemia	74 (24.7%)	9 (16.4%)	28 (39.4%)	25 (25%)	6 (26.1%)	6 (11.8%)	0.005
Marsh 3b/3c^b^	89 (61.8%)	18 (75%)	17 (74%)	28 (50%)	4 (50%)	22 (67%)	0.125

^a^*AI* Autoimmune

^b^Only 144 patients underwent duodenal biopsy: 24 patients of G1 class, 23 of G2, 56 of G3, 8 of G4, 33 of G5

Only 38 patients were asymptomatic, 8 of which from G1 class, 7 from G2, 17 from G3, 1 from G4 and 5 from G5. The other 262 (87.3%) patients had heterogeneous gastrointestinal and extraintestinal symptoms. Although, in all classes diarrhea occurred more than constipation, comparing G1 and G5 class, we found a relevant significance (*p* = 0.046) between the frequency of diarrhea in the G1 and G5 (*n* = 26; 47% vs *n* = 14; 27% respectively) We also found a difference in constipation, that occurred more frequently in G5 class (*n* = 11; 22%) and rarely in G1 (*n* = 6; 11%), although this latest association was not statistically significant (*p* = 0.135). In 97 patients (32.3%) clinical history described an atopic syndrome and G5 showed the highest frequency (*n* = 19; 37,3%), while G2 the lowest frequency (*n* = 19; 27%) with a *p*-value = 0.779, not statistically significant. Only in 33 patients CD was present simultaneously with type I DM and/or thyroid disease, and the largest population belonged to G5 class (*n* = 9; 17.6%), while the smallest population belonged to G4 class (*n* = 1; 4%), although this association was not statistically significant (*p* = 0.664). We observed a disparity in the severity of the villous lesion among the classes: G1 class patients’ biopsy showed a severe lesion (Marsh 3b-3c) in 75% (*n* = 18) of cases, G2 class in 74% (*n* = 17), G3 and G4 classes only in 50% (*n* = 28 vs *n* = 4 respectively) and G5 class in 67% (*n* = 22), but this relationship was not statistically significant (*p* = 0.125). Instead, in 194 patients (64.7%) levels of tTG IgA were ≥ 100 U/mL and the highest frequency (*n* = 44; 80%; *n* = 16; 69.6%; *n* = 48; 67.6%) belonged to G1, G4 and G2 group respectively, and the association between antibody levels and HLA class risk was statistically significant (*p* = 0.037). Finally, there was a statistically significant difference among the risk classes’ levels in terms of enhanced liver enzymes. Indeed, an isolated hypertransaminasemia was detected in 74 patients (24.7%) and interestingly G2 showed the highest frequency (*n* = 28; 39.4%, *p* = 0.005). Results from multiple logistic regression showed that, after adjusting for the effect of gender, age at onset and family history, HLA class risk was still significantly associated with anti-tTG ≥ 100 (*p* = 0.044) and with hypertransaminasemia (*p* = 0.010).

## Discussion

In literature it has been widely described that genetic susceptibility and environmental factors can influence celiac disease clinical manifestations. It is also known that genetic susceptibility, essential to the onset of disease, is given by HLA-DQ haplotypes but how genetic background modules celiac disease is still not clear [17–21]. Indeed, it is still unknown the relationship between HLA genetics and CD phenotype, and some authors relate HLA genetics only with some clinical data but not others [20–25]. Whereas, we have previously reported also the influence of non-HLA genes on CD phenotype [26]. We present in this retrospective observational study the experience of the Pediatric Gastroenterology Department of University of Campania “Luigi Vanvitelli” with the aim of evaluating the possible influence of HLA-DQ genotypes on the clinical, analytical and histological manifestations at the onset of CD, estimating differences among the five HLA-DQ risk classes. As commonly reported in pediatric series with CD [27–29] we found a predominance in girls and early onset, which was also associated to classical clinical presentation. Instead, older age of onset was significantly associated with the coexistence of other autoimmune diseases.

Moreover, we found an increased frequency of atopy in male CD which showed an increased IgE sensitization. Although it is well known that the two diseases don’t share common pathogenic pathways, a mechanism behind this possible association might be an increased intestinal permeability in individuals with CD resulting in increased flow of dietary antigens [30, 31], that could lead to increased IgE sensitization. Other possible reasons for this association could be dysregulation of immune responses or common genetics.

The Dieterich paper [32] demonstrates that gliadin is the preferred substrate of transglutaminase suggesting that the interaction of gliadin and transglutaminase may result in the creation of new antigenic complexes. These neoepitopes were bound to antigen-presenting cells and presented to T cells in the gut. While in celiac disease activated T cells CD4+ start producing mainly TH1 cytokines, as IFN-γ, in the atopic syndrome TH2 cytokines play the most important role. On the other hand, regulatory T (T-reg) cells, both “natural” forkhead box protein 3 T-reg cells and “induced” T-reg cells, the latter producing IL-10, have been implicated in the control of both TH1 along with TH2 responses [31]. However, it has been identified a T-reg cells’ dysfunction in patients suffering from atopic syndrome [33].

Another reason behind the association between CD and atopy (in particular asthma) may be malnutrition, because in about 60 to 70% of celiac patients, laboratory tests even years after diagnosis show low levels of 25-(OH) vitamin D [34]. In fact, vitamin D plays an important role in immune system’s regulation: calcitriol can act on T-reg cells directly, inhibiting proliferation and inducing IL-2 production, or indirectly, leading T-reg cells to promote its effect, but it can also regulate immune system acting on dendritic cells directly or indirectly [35]. Therefore, low levels of vitamin D as described in CD, could generate T-reg cells unable to control and suppress T-cells responses contributing to the onset of atopy. Finally, some authors hypothesize a shared immunological pathway due to IL-15, that is indeed involved in both asthma and CD [36–39].

Regarding the association of HLA-DQ genotypes, we found that patients belonging to G1, G4 and G2 class had significantly higher tTG IgA levels, confirming a gene-dose effect of the DQB1–02 allele on anti-transglutaminase antibodies levels in CD as previously described [40]. Indeed, HLA-molecules are fundamental to determine CD4+ T-cells activation, resulting in the further activation of other immune cells, including B-cells [41–43]. Thus, an increased number of CD-associated heterodimers expressed on cell surface might be responsible for an increased antigen presentation, and a consequent T- and B-cell stimulation, with a stronger antibody response. We observed also an association between DQB1–02 alleles and symptoms, finding that a typical clinical presentation with diarrhoea was increased in carriers of HLA-DQ2.5 with double HLADQB1* 02 dose. A similar effect was underlined by Zubillaga et al. [20] and Piccinni et al. [25], the last ones describing higher frequency of atypical or silent/latent CD in patients with low genetic risk. Differently from other studies [22, 24], we did not find a significant association of HLA risk classes with severity of mucosal lesion, and in accordance with the results of our previous study we hypothesized a role for non-HLA genes to explain this histological data [26]. Moreover, only half of the patients underwent duodenal biopsies which could underestimate the gene dose effect in this context reducing the significance of our data.

Interestingly we found an association between G2 and hypertransaminasemia. To note in the G2 group we also found higher tTG Ab titers and consequent villous atrophy. Accordingly, both in adults [44] and in children [45] it has been reported increased ALT to be associated with more high autoantibody levels and severe villous atrophy. Malabsorption may play a role to explain hypertransaminasemia, [46, 47] as well as the alteration of intestinal permeability with a “leaky” intestine [48]. In fact, toxins coming from food could be able to reach more easily the liver via the portal circulation, causing a hepatic inflammatory state, as demonstrated on patients’ liver biopsies [49]. This hypothesis has been strengthened by Novacek et al. [50], that, using the urinary recovery methods of sugars, found an association between serum transaminase level and permeability index.

Finally, it has been proposed also a direct effect of tTG antibodies on liver transglutaminase [51, 52]. This ubiquitous enzyme has a protective effect on liver injury [53] and this protective effect may be affected by the presence of antibodies to tTG, [44] that have been described in the duodenum, but also in the liver [54] and nervous system [55]. To the best of our knowledge we found for the first time an association between HLA- DQ2 and hypertransaminasemia, which suggest that also liver damage in CD could be related to HLA haplotype. Given the diagnostic applicability of HLA Typing our results suggest its possible role also in risk stratification. Early identification of high-risk patients would be of utmost importance. Indeed, it would be useful the design of accurate and tailored CD follow up strategies according to the haplotype of the patient. A closer follow-up and a stricter gluten-free diet might help them to avoid the development of life-threatening complications (e.g., liver damage, malignancies) [45, 56, 57].

Our main strengths are the well-defined and large cohort of celiac patients, who were diagnosed according to harmonized nationwide guidelines in the same centre and revised by the same physician. Therefore, no bias by different clinical practice exists. Limitations of our study are inherent to the retrospective study and the utilization of self-reported family history and symptoms of CD, although the majority of information was available in the medical record. Also, all our study subjects were with Italian ancestry, which may limit the generalizability to other study settings with a different ethnic composition.

Finally, genetic analysis was also limited to the assessment of the frequency of known celiac disease HLA risk haplotypes, and thus no deeper insight into the role of non-HLA genes and gene-to-gene interactions could be attained.

## Conclusions

In conclusion, we failed to prove an association between HLA-DQ genotypes and the clinical features. Although, our results suggest an effect of the DQB1–02 allele not only on the level of antibodies to tTG, but possibly also on liver involvement.

It may be that differences also exist between CD patients with HLA-DQ2.5 with single dose and those carrying HLA-DQ8 or lower risk HLA genotypes. The frequency of patients with these genetics is very low, and a multicenter study would be necessary to address these haplotypes’ role.

## Data Availability

The datasets used and analysed during the current study are available from the corresponding author on reasonable request.

## Abbreviations

CD: Celiac disease
tTG: Tissue Transglutaminase
DM: Diabetes Mellitus
EMA: Endomysial antibody
IFN-γ: Interferon-γ
T-reg cells: T-regulatory cells

## References

[1] Mäki M, Collin P (1997). Coeliac disease. Lancet.

[2] Catassi C, Kryszak D, Louis-Jacques O, Duerksen DR, Hill I, Crowe SE, Brown AR, Procaccini NJ, Wonderly BA, Hartley, M.D. P, Moreci J, Bennett N, Horvath K, Burk M, Fasano A (2007). Detection of celiac disease in primary care: a multicenter case-finding study in North America. Am J Gastroenterol.

[3] Alshiekh S, Zhao LP (2017). Different DRB1*03:01-DQB1*02:01 haplotypes confer different risk for celiac disease. HLA.

[4] Fernandez-Jimenez N, Bilbao J.R., Bilbao JR Mendelian randomization analysis of celiac GWAS reveals a blood expression signature with diagnostic potential in absence of gluten consumption. Hum Mol Genet 2019; 28(18):3037–3042, DOI: 10.1093/hmg/ddz113.10.1093/hmg/ddz113PMC673729131127932

[5] Taylor AK, Lebowhl B (2008). Celiac disease. GeneReviews.

[6] Sollid LM, Jabri B (2013). Triggers and drivers of autoimmunity: lessons from coeliac disease. Nat Rev Immunol.

[7] Tolone C, Cirillo G, Papparella A, Tolone S, Santoro N, Grandone A, Perrone L, del Giudice EM (2009). A common CTLA4 polymorphism confers susceptibility to autoimmune thyroid disease in celiac children. Dig Liver Dis.

[8] Maltoni G, Franceschi R (2017). Prevalence of celiac disease in 52, 721 youth with type 1 diabetes: international comparison across three continents. Diabetes Care.

[9] Anania C, De Luca E (2015). Liver involvement in pediatric celiac disease. World J Gastroenterol.

[10] Roy A, Laszkowska M, Sundström J, Lebwohl B, Green PHR, Kämpe O, Ludvigsson JF (2016). Prevalence of celiac disease in patients with autoimmune thyroid disease: a meta-analysis. Thyroid.

[11] Hill ID, Dirks MH, Liptak GS, Colletti RB, Fasano A, Guandalini S, Hoffenberg EJ, Horvath K, Murray JA, Pivor M, Seidman EG, North American Society for Pediatric Gastroenterology, Hepatology and Nutrition (2005). Guideline for the diagnosis and treatment of celiac disease in children: recommendations of the north American Society for Pediatric Gastroenterology, Hepatology and nutrition. J Pediatr Gastroenterol Nutr.

[12] ESPGHAN (2020). Guidelines for diagnosing coeliac disease.

[13] Margaritte-Jeannin P, Babron MC, Bourgey M, Louka AS, Clot F, Percopo S, Coto I, Hugot JP, Ascher H, Sollid LM, Greco L, Clerget-Darpoux F (2004). HLA-DQ relative risks for coeliac disease in European populations: a study of the European genetics cluster on coeliac disease. Tissue Antigens.

[14] ESPGHAN (2012). Guidelines for diagnosing coeliac disease.

[15] Walker M, Murray J (2010). An update in the diagnosis of celiac disease. Histopathology.

[16] Bourgey M, Calcagno G (2007). HLA related genetic risk for coeliac disease. Gut.

[17] Ploski R, Ek J, Thorsby E, Sollid LM (1993). On the HLA-DQα1, β1-associated susceptibility in celiac disease: a possible gene dosage effect of DQB1_0201. Tissue Antigens.

[18] Congia M, Cucca F, Frau F, Lampis R, Melis L, Clemente MG, Cao A, de Virgiliis S (1994). Gene dosage effect of the DQA1_0501/DQB1_0201 allelic combination influences the clinical heterogeneity of celiac disease. Hum Immunol.

[19] Greco L, Percopo S, Clot F, Bouguerra F, Babron MC, Eliaou JF, Franzese C, Troncone R, Clerget-Darpoux F (1998). Lack of correlation between genotype and phenotype in celiac disease. J Pediatr Gastroenterol Nutr.

[20] Zubillaga P, Vidales MC, Zubillaga I, Ormaechea V, García-Urkía N, Vitoria JC (2002). HLA-DQA1 and HLADQB1 genetic markers and clinical presentation in celiac disease. J Pediatr Gastroenterol Nutr.

[21] Karinen H, Ka¨rkka¨inen P, Pihlajama¨ki J, et al. (2006). Gene dose effect of the DQB1_0201 allele contributes to severity of coeliac disease. Scand J Gastroenterol.

[22] Jores RD, Frau F, Cucca F, Grazia Clemente M, Orrù S, Rais M, de Virgiliis S, Congia M (2007). HLADQB1*0201 homozygosis predisposes to severe intestinal damage in celiac disease. Scand J Gastroenterol.

[23] Liu E, Lee HS, Aronsson CA, Hagopian WA, Koletzko S, Rewers MJ, Eisenbarth GS, Bingley PJ, Bonifacio E, Simell V, Agardh D, TEDDY Study Group (2014). Risk of pediatric celiac disease according to HLA haplotype and country. N Engl J Med.

[24] Nenna R, Mora B, Megiorni F, Mazzilli MC, Magliocca FM, Tiberti C, Bonamico M (2008). HLA-DQB1*02 dose effect on RIA anti-tissue transglutaminase autoantibody levels and clinicopathological expressivity of celiac disease. J Pediatr Gastroenterol Nutr.

[25] Piccini B, Vascotto M, Serracca L, Luddi A, Margollicci MA, Balestri P, Vindigni C, Bassotti G, Villanacci V (2012). HLA-DQ typing in the diagnostic algorithm of celiac disease. Rev Esp Enferm Dig.

[26] Galatola M, Izzo V, Cielo D, Morelli M, Gambino G, Zanzi D, Strisciuglio C, Sperandeo MP, Greco L, Auricchio R. Gene expression profile of peripheral blood monocytes: a step towards the molecular diagnosis of celiac disease? PLoS One. 2013;8(9):e74747. 10.1371/journal.pone.0074747.10.1371/journal.pone.0074747PMC377574524069342

[27] Cilleruelo ML, Roman-Riechmann E, Sanchez-Valverde F, Donat E, Manuel-Ramos J, Martín-Orte E, López MJ, García-Novo D, García S, Pavón P, Martín M, Ortigosa L, Barrio J, Gutierrez C, Espìn B, Castillejo G, Peña-Quintana L, Hualde I, Sebastián M, Calvo C, Fernández S, de Manueles J, Armas H, Urruzuno-Tellerias P, Juste M, Bousoño C, Ribes-Koninckx C (2014). Spanish national registry of celiac disease: incidence and clinical presentation. J Pediatr Gastroenterol Nutr.

[28] Llorente-Alonso MJ, Fernandez-Acenero MJ, Sebastian M (2006). Gluten intolerance: sex and age-related features. Can J Gastroenterol.

[29] Misak Z, Hojsak I, Jadresin O (2013). Diagnosis of coeliac disease in children younger than 2 years. J Pediatr Gastroenterol Nutr.

[30] Pillon R, Ziberna F, Badina L, Ventura A, Longo G, Quaglia S, de Leo L, Vatta S, Martelossi S, Patano G, Not T, Berti I (2015). Prevalence of celiac disease in patients with severe food allergy. Allergy.

[31] Ludvigsson JF, Hemminki K, Wahlström J, Almqvist C (2011). Celiac disease confers a 1.6-fold increased risk of asthma: a nationwide population-based cohort study. J Allergy Clin Immunol.

[32] Dieterich W, Ehnis T, Bauer M, Donner P, Volta U, Riecken EO, Schuppan D (1997). Identification of tissue transglutaminase as the autoantigen of celiac disease. Nat Med.

[33] Robinson DS (2009). Regulatory T cells and asthma. Clin Exp Allergy.

[34] Hallert C, Grant C, Grehn S (2002). Evidence of poor vitamin status in coeliac patients on a gluten-free diet for 10 years. AlimentPharmacol Ther.

[35] Dimeloe S, Nanzer A, Ryanna K, Hawrylowicz C (2010). Regulatory T cells, inflammation and the allergic response-the role of glucocorticoids and vitamin D. J Steroid Biochem Mol Biol.

[36] Nishiwaki T, Ina K, Goto H, Watanabe O, Tsuzuki T, Furuta R, Ando T, Hibi K, Kusugami K (2005). Possible involvement of the interleukin-15 and interleukin-15 receptor system in a heightened state of lamina propria B cell activation and differentiation in patients with inflammatory bowel disease. J Gastroenterol.

[37] Mori A, Suko M, Kaminuma O (1996). IL-15 promotes cytokine production of human T helper cells. J Immunol.

[38] Kurz T, Strauch K, Dietrich H, Braun S, Hierl S, Jerkic SP, Wienker TF, Deichmann KA, Heinzmann A (2004). Multilocus haplotype analyses reveal association between 5 novel IL-15 polymorphisms and asthma. J Allergy Clin Immunol.

[39] Meresse B, Chen Z, Ciszewski C, Tretiakova M, Bhagat G, Krausz TN, Raulet DH, Lanier LL, Groh V, Spies T, Ebert EC, Green PH, Jabri B (2004). Coordinated induction by IL15 of a TCR-independent NKG2D signaling pathway converts CTL into lymphokine-activated killer cells in celiac disease. Immunity..

[40] Mubarak A, Spierings E, Wolters VM, Otten HG, ten Kate F, Houwen RH (2013). Children with celiac disease and high tTGA are genetically and phenotypically different. World J Gastroenterol.

[41] Lundin KE, Scott H, Hansen T, Paulsen G, Halstensen TS, Fausa O, Thorsby E, Sollid LM (1993). Gliadin-specific, HLA-DQ (alpha 1*0501,beta 1*0201) restricted T cells isolated from the small intestinal mucosa of celiac disease patients. J Exp Med.

[42] Osman AA, Günnel T, Dietl A, Uhlig HH, Amin M, Fleckenstein B, Richter T, Mothes T (2000). B cell epitopes of gliadin. Clin Exp Immunol.

[43] Vader W, Stepniak D, Kooy Y, Mearin L, Thompson A, van Rood JJ, Spaenij L, Koning F (2003). The HLA-DQ2 gene dose effect in celiac disease is directly related to the magnitude and breadth of gluten-specific T cell responses. Proc Natl Acad Sci U S A.

[44] Zanini B, Baschè R, Ferraresi A, Pigozzi MG, Ricci C, Lanzarotto F, Villanacci V, Lanzini A (2014). Factors that contribute to hypertransaminasemia in patients with celiac disease or functional gastrointestinal syndromes. Clin Gastroenterol Hepatol.

[45] Äärelä L, Nurminen S, Kivelä L, Huhtala H, Mäki M, Viitasalo A, Kaukinen K, Lakka T, Kurppa K (2016). Prevalence and associated factors of abnormal liver values in children with celiac disease. Dig Liver Dis.

[46] Etukudo MH, Agbedana EO, Akinyinka OO, Osifo BO (1999). Plasma electrolytes, total cholesterol, liver enzymes, and selected antioxidant status in protein energy malnutrition. Afr J Med Med Sci.

[47] Hanachi M, Melchior JC, Crenn P (2013). Hypertransaminasemia in severely malnourished adult anorexia nervosa patients: risk factors and evolution under enteral nutrition. Clin Nutr.

[48] Smecuol E, Bai JC, Vazquez H, Kogan Z, Cabanne A, Niveloni S, Pedreira S, Boerr L, Maurino E, Meddings JB (1997). Gastrointestinal permeability in celiac disease. Gastroenterology.

[49] Foley A, Sheperd SJ, Gibson PR (2010). Frequency of elevated ALT in untreated coeliac disease and the impact of compliance with gluten free diet on ALT normalisation. Gastroenterology.

[50] Novacek G, Miehsler W, Wrba F, Ferenci P, Penner E, Vogelsang H (1999). Prevalence and clinical importance of hypertransaminasemia in coeliac disease. Eur J Gastroenterol Hepatol.

[51] Pelaez-Luna M, Schmulson M, Robles-Diaz G (2005). Intestinal involvement is not sufficient to explain hypertransaminasemia in celiac disease?. Med Hypotheses.

[52] Sainsbury A, Sanders DS, Ford AC (2011). Meta-analysis: coeliac disease and hypertransaminasemia. Aliment Pharmacol Ther.

[53] Aeschlimann D, Paulsson M (1991). Cross-linking of laminin-nidogen complexes by tissue transglutaminase. A novel mechanism for basement membrane stabilization. J Biol Chem.

[54] Korponay-Szabo IR, Halttunen T, Szalai Z (2004). In vivo targeting of intestinal and extraintestinal transglutaminase 2 by coeliac autoantibodies. Gut.

[55] Hadjivassiliou M, Maki M, Sanders DS, Williamson CA, Grunewald RA, Woodroofe NM, Korponay-Szabo IR (2006). Autoantibody targeting of brain and intestinal transglutaminase in gluten ataxia. Neurology.

[56] Megiorni F, Pizzuti A (2012). HLA-DQA1 and HLA-DQB1 in celiac disease predisposition: practical implications of the HLA molecular typing. J Biomed Sci.

[57] Romanos J, van Diemen CC, Nolte IM, Trynka G, Zhernakova A, Fu J, Bardella MT, Barisani D, McManus R, van Heel DA, Wijmenga C (2009). Analysis of HLA and non-HLA alleles can identify individuals at high risk for celiac disease. Gastroenterology..

